# Prediction Models for Return of Spontaneous Circulation in Patients with Cardiac Arrest: A Systematic Review and Critical Appraisal

**DOI:** 10.1155/2023/6780941

**Published:** 2023-11-21

**Authors:** Pengfei Cheng, Pengyu Yang, Hua Zhang, Haizhen Wang

**Affiliations:** ^1^Department of Nursing, Second Affiliated Hospital of Zhejiang University, Hangzhou 310009, China; ^2^School of International Nursing, Hainan Medical University, Haikou 571199, China; ^3^Key Laboratory of Emergency and Trauma Ministry of Education, Hainan Medical University, Haikou 571199, China

## Abstract

**Objectives:**

Prediction models for the return of spontaneous circulation (ROSC) in patients with cardiac arrest play an important role in helping physicians evaluate the survival probability and providing medical decision-making reference. Although relevant models have been developed, their methodological rigor and model applicability are still unclear. Therefore, this study aims to summarize the evidence for ROSC prediction models and provide a reference for the development, validation, and application of ROSC prediction models.

**Methods:**

PubMed, Cochrane Library, Embase, Elsevier, Web of Science, SpringerLink, Ovid, CNKI, Wanfang, and SinoMed were systematically searched for studies on ROSC prediction models. The search time limit was from the establishment of the database to August 30, 2022. Two reviewers independently screened the literature and extracted the data. The PROBAST was used to evaluate the quality of the included literature.

**Results:**

A total of 8 relevant prediction models were included, and 6 models reported the AUC of 0.662–0.830 in the modeling population, which showed good overall applicability but high risk of bias. The main reasons were improper handling of missing values and variable screening, lack of external validation of the model, and insufficient information of overfitting. Age, gender, etiology, initial heart rhythm, EMS arrival time/BLS intervention time, location, bystander CPR, witnessed during sudden arrest, and ACLS duration/compression duration were the most commonly included predictors. Obvious chest injury, body temperature below 33°C, and possible etiologies were predictive factors for ROSC failure in patients with TOHCA. Age, gender, initial heart rhythm, reason for the hospital visit, length of hospital stay, and the location of occurrence in hospital were the predictors of ROSC in IHCA patients.

**Conclusion:**

The performance of current ROSC prediction models varies greatly and has a high risk of bias, which should be selected with caution. Future studies can further optimize and externally validate the existing models.

## 1. Introduction

Cardiac arrest (CA) is an enormous public health issue all over the world. Despite years of effort, the discharge survival rate of CA patients remains unfavorable [1]. In the United States, out-of-hospital cardiac arrest (OHCA) affects more than 88.8/100,000 adults annually, according to a report by the American Heart Association (AHA) [2]. The risk of in-hospital cardiac arrest (IHCA) was greater (17.16/1000), whereas the rate of discharge survival was only 9.0% and 23.3%, respectively. In an analogous manner, the yearly incidence of OHCA in adults in Europe is from 67/100,000 to 170/100,000 , whereas the incidence of IHCA is from 1.5/1000 to 2.8/1000 . The survival rates at the time of discharge ranged from 0 to 18% and, correspondingly, 15% to 34% [3]. The return of spontaneous circulation, often known as ROSC, is an essential indication that is utilized in the evaluation of early vital signs in patients who have CA. It not only represents the immediate effectiveness of initial resuscitation in IHCA patients but also the influence of cardiopulmonary resuscitation (CPR) on the survival of OHCA patients [4–6]. For this reason, it is an important reference and impact on the subsequent implementation of advanced life support (ALS) and patient discharge survival rate to accurately predict the ROSC probability of CA patients [7, 8]. The ROSC prediction model can also assist medical professionals in assessing the status and likelihood that patients will survive after resuscitation in nations and regions with scarce emergency resources, allowing for the best possible resuscitation outcomes with the least amount of resource expenditure [9]. Simultaneously, in order to avoid ambiguity and disagreement in the area of moral management of cardiac arrest patients who have refractory cardiac arrest and to uphold patients' final dignity, it is helpful for medical professionals to better determine the timing and standard of termination of resuscitation (TOR) [10]. Although several research studies had been conducted on ROSC prediction models, there are still significant discrepancies in literature quality, model performance, predicators, and application breadth. Therefore, we aimed to systematically review and critically evaluate all the current prediction models for ROSC and give a reference for clinical practice as well as for upcoming research.

## 2. Methods

### 2.1. Systematic Review Registration

Before data extraction, this review (CRD42022331873) was registered and made public with PROSPERO (the international prospective register of systematic reviews).

### 2.2. Search Strategy

Following the preferred reporting items for systematic reviews and meta-analyses (PRISMA) recommendations [11], we conducted an electronic literature search of PubMed, Cochrane Library, Embase, Elsevier, Web of Science, SpringerLink, Ovid, China National Knowledge Internet (CNKI), Wanfang database, and Chinese Biomedical literature database (SinoMed). Also, we included literature published from inception until 1 August 2022, using a mix of subject headings that includes “cardiac arrest”/“restoration of autonomic circulation”/“predictive model”/“risk score.” The references of all the publications that the search turned up were then carefully checked. Considering the PubMed search formula as an example was as follows: (“Return of Spontaneous Circulation”(MeSH)) AND (“Heart Arrest”(MeSH) OR “Cardiopulmonary Resuscitation”(MeSH) OR “Cardiac Arrest”(Title/Abstract)) AND (“predict^*∗*^”(Title/Abstract) OR “risk prediction”(Title/Abstract) OR “risk score”(Title/Abstract) OR “risk assessment”(Title/Abstract)) AND (“model”(Title/Abstract) OR “score”(Title/Abstract)).

### 2.3. Study Eligibility Criteria

Inclusion criteria were as follows: (1) the study's participants were cardiac arrest patients over the age of 18; (2) the development of ROSC prediction models, including models for both success and failure in ROSC; and (3) cohort studies, case-control studies, or cross-sectional studies were the three research types used.

Exclusion criteria were as follows: (1) only impact factor studies that did not build prediction models would be eliminated; (2) conference abstracts, reviews, commentaries, and relevant data were seriously missing in the literature; (3) cellular-molecular level studies and animal experimental studies; (4) full text was not available; and (5) less than two predictor variables were present in the model.

### 2.4. Study Selection and Data Extraction

Title, abstract, and full-text articles of the retrieved papers were separately reviewed by two researchers. Conflicts were settled amicably with the help of a third reviewer. Following the discovery of the included literature, data from the included studies were systematically extracted using the criteria of the checklist for critical appraisal and data extraction for systematic reviews of prediction modeling studies checklist (CHARMS checklist) [12]. This checklist includes details about the year, nation (or region), design, object, data source, ROSC rate, results, sample size, missing data, candidate predictors' number, variable selection, modeling method, testing method, model performance, predictors in the final model, applicability, and limitations.

### 2.5. Assessment of Bias Risk and Applicability

The two researchers used the Prediction Model Risk of Bias ASsessment Tool (PROBAST) [13], which was created expressly to evaluate diagnostic and prognostic prediction models, to evaluate the risk of bias and application of the literature that had been gathered. The tool's risk of bias evaluation contains the following four aspects: participants, predictors, outcome, and analysis, with the applicability assessment mostly focused on participants, predictors, and outcome.

### 2.6. Statistical Evaluation

The metagen command of meta-analysis package in R statistical language software (v 4.1.3) was used to perform meta-analysis on the sensitivity, specificity, AUC, and 95% CI of the included model in development and validation data. We used the between-study standard deviation (tau-*τ*) and *I*^2^ statistic to quantify possible heterogeneity among the studies. If there was large heterogeneity among the studies, the random-effect model was used for the combined analysis. If the heterogeneity among the studies was small, the fixed-effect model was used for the pooled analysis.

## 3. Results

### 3.1. Study Selection

Figure 1 depicts the process of doing literature research and selecting studies. By combing through databases and following citations by hand, we were able to compile a list of 5691 related articles. After screening, a total of 8 papers meeting the criteria were finally included.

### 3.2. Study Characteristics

Table 1 shows the basic characteristics of the ROSC prediction model studies included in the systematic review. Among the eight studies [14–21] finally included, four [14, 15, 20, 21] were retrospective cohort studies, two [17, 18] were prospective cohort studies, and two [16, 19] were retrospective case-control studies. Half of these studies (*n* = 4) [14, 15, 18, 19] were conducted in Europe, and four [16, 17, 20, 21] in Asia. Interestingly, all but one study [15] used IHCA as the study subject, while all other studies used OHCA as the study subject. Seven studies [14–19, 21] used ROSC success as an outcome indicator, and only one study [20] was conducted with ROSC failure as an outcome indicator, that is, ROSC could not be achieved after continuous resuscitation.

### 3.3. Severity Prediction

Each study's sample size for model development ranged from 347 to 119,474 instances, and the number of possible predictor variables ranged from 7 to 14, all of which were addressed with absolute exclusion for missing data cases. Only one study [21] ranked the significance of candidate predictors based on the results of logistic regression and included the top 5 ranked factors as predictor variables. Five studies [14, 16, 18–20] adopted the screening of predictors based on the results of single factor analysis, and two studies [15, 17] directly used the stepwise selection method of multifactor analysis. Regarding the development of prediction models, the modeling method used most frequently in these models [14, 15, 17, 18, 20] was logistic regression, and Cox proportional hazard regression was also used in one model [16]. There were also mixed-effects regression [19] and machine learning [21] modeling approaches for these models but only one study each.

### 3.4. Model Performance and Predictors

Of all the models included, eight [14–21] were internally validated and one-third of the models (*n* = 3; 37.5%) [15, 18, 20] had external validation. As for the performance of the prediction model, AUC (area under the receiver operating characteristic curve) of the model was reported by six studies [14, 17–21], and Harrison et al. [15] evaluated the model's differentiation with the concordance index (C-index). Kim et al. [16] did not elaborate on this in their study. Three studies [15, 16, 19] adopted reasonable inspection methods to evaluate the calibration degree of the model and reported the calibration results of the model. In addition, only Amnuaypattanapon et al. [17], Baldi et al. [18], and Kuo et al. [20] had fully explained the sensitivity and specificity of the model (Table 1).

Most models [14, 16–19, 21] were established with OHCA patients as research objects. The most common candidate predictors were initial heart rhythm (frequency ≥2), etiology, age, location, bystander CPR, witnessed at arrest, EMS arrival time, sex, and time of BLS (Figure 2). The main predictors of ROSC in IHCA patients, according to Gräsner et al. [14], were age, gender, length of hospital stay, medical reasons, location of cardiac arrest, and initial heart rhythm. The presence of apparent chest injury, a temperature less than 33 degrees Celsius, and a probable etiology of OHCA were all variables that could predict ROSC failure in traumatic out-of-hospital cardiac arrest (TOHCA) patients [20].

### 3.5. Risk of Bias and Applicability

#### 3.5.1. Domain 1: Participants

Since the majority of the study's data sources were cohort studies, there is a minimal risk of bias in the participant selection criteria; nevertheless, there are still two studies [16, 20] with a high risk of bias. For example, the study by Kim et al. [16] and another study by Kuo et al. [20] both were retrospective and the data were, respectively, from the emergency department of a hospital in Seoul, Korea, and a trauma medical center in Taiwan, China. Because the data sources were not randomized controlled designs, registry databases, or prospective cohort studies as indicated by PROBAST low bias criteria, the participants in the research were found to be at a high risk of bias.

#### 3.5.2. Domain 2: Predictors

All of the studies included in this systematic review had a bias in the predictors' domain, which was mainly a low concern for risk.

#### 3.5.3. Domain 3: Outcome

Of all the studies, most were considered to be a low risk of bias in the outcome domain (*n* = 5, 62.5%); [14–17, 20] what was interesting was that the remaining three studies [18, 19, 21] were also classified as low bias in all other aspects of consequence evaluation, but the total rating was unclear in the outcome domain. Unclear items focus primarily on the researchers who did not know if the interval between predictor assessment and outcome determination was appropriate. Due to the absence of these two components in the three studies, knowledge of predictor outcomes may impact the determination and cause bias.

#### 3.5.4. Domain 4: Analysis

Within the domain of analysis, every study was assigned a high level of concern for risk. Eight studies [14–21] had sufficient data sources, both in terms of the sample size to meet the fundamental requirements of the model building and validation, and handling of continuous variables was also consistent with two or more categories but not consistent when dealing with the missing value to take multiple methods of interpolation to directly rule out missing data; this method was very simple but may be associated with a high risk of bias, so the 8 studies were included. In addition, 5 studies [14, 16, 18–20] adopted the method of screening predictors based on the results of single factor analysis, which was also highly biased. In terms of the calibration degree of the model, Kim et al. [16] used Grønnesby and Borgan goodness of fit tests to measure the calibration degree of the model. Harrison et al. [15] and Ji et al. [19] used the Hosmer–Lemeshow test, Cox calibration, calibration plot, and Brier scores to evaluate the calibration degree and fit of the model. However, other 5 studies [14, 15, 18, 20, 21] had insufficient information.

### 3.6. Applicability

Table 2 displays the results of the bias risk assessment contained in the mode (PROBAST evaluation results). As you can see, all of the included studies' models performed well in the domains of participants, predictors, and outcomes, as well as the overall evaluation.

### 3.7. Meta-Analysis of Prediction Models

The AUC of the included models were reported in 6 studies [14, 17–21], of which 4 [14, 18, 19, 21] detailed the AUC of the models on the validation data, so we conducted a meta-analysis of AUC in the 11 data to maximize the sample size. Considering the large heterogeneity (*I*^2^ = 99%) after data synthesis, the random-effect model was used, and the results of meta-analysis showed that the pooled AUC was 0.74 (95% CI: 0.71–0.78) (Figure 3). In addition, only 3 of the included studies had sensitivity and specificity of the model [17, 18, 20], of which 1 study [20] lacked 95% CI, so we only synthesized the other 2 [17, 18]. The results of meta-analysis showed that the heterogeneity was *I*^2^ = 96%, the pooled sensitivity was 0.60 (95% CI: 0.42–0.87) (Figure 4), and pooled specificity was 0.84 (95% CI: 0.69–1.03) (Figure 5).

## 4. Discussion

### 4.1. Overall Situation of the ROSC Prediction Model

A high-quality prediction model can effectively and accurately reflect ROSC of patients with CA, which gives significant reference values to subsequent clinical decision-making and medical resource applications. The AUC or C-index of the models involved in the eight studies [14–21] finally included in this paper were all lower than 0.90 and the pooled AUC was 0.74 (95% CI: 0.71–0.78), which means that the ROSC prediction models constructed by most current studies have a certain degree of discrimination for the prediction of ROSC in patients with cardiac arrest, but the discrimination ability was only at the medium level. According to the results of meta-analysis, the pooled sensitivity and specificity were 0.60 (95% CI: 0.42–0.87) and 0.84 (95% CI: 0.69–1.03), respectively, indicating that the current ROSC prediction model has high specificity and low sensitivity in terms of accuracy, and there were still insufficient to achieve desired high accurate prediction. In addition, all prediction models were rated as high-risk bias by PROBAST. The bias was mainly attributed to retrospective research, missing value processing, variable screening, model validation, model performance evaluation, and overfitting, among which missing value processing was a widespread problem in all studies. Since the data of most researchers were directly obtained from OHCA or IHCA registration database based on the Utstein model, a sufficient sample size was guaranteed for model construction and verification. Hence, the method of direct exclusion was adopted when processing initial values, which might lead to the omission of effective information, reduce the accuracy of model prediction, and cause bias in analysis results [22]. As for the screening of predictors, there were five studies [14, 16, 18–20] based on univariate analysis. However, univariate analysis usually fails to identify the interaction between confounding factors and variables due to its statistical limitations, even leading to the omission of important risk factors. Therefore, the variable screening method based on univariate analysis is not recommended in the future logistic model or nomogram model construction. Instead, the potential bias risk can be reduced by using the full inclusion method and Lasso regression analysis to screen variables [23]. In addition, all the included studies did not make comprehensive and detailed reports on model validation, model performance evaluation, and overfitting and lacked a full explanation of the transparency of the overall research and the limitations of the prediction model, which led to doubts on the authenticity and reliability of the model and thereby hindered the universal application and external promotion of the prediction model.

### 4.2. Models to Predict Outcome Events

Almost all of the included studies took ROSC as the outcome event, except for the study conducted by Kuo et al. [20] that used ROSC failure as the outcome event to explore the important risk factors of TOHCA so as to help clinical doctors and nurses complete the assessment of priority resuscitation in the shortest time when managing multiple patients with severe traumatic sudden arrest at the same time. Although most models use sustained ROSC as the outcome event, there are still differences in the definition of sustained ROSC in different studies. Gräsner et al. [14] defined sustained ROSC as that the patient's pulse recovers and is accessible for more than 20 s, while Amnuaypattanapon et al. [17] defined sustained ROSC as that after the patient is resuscitated, the circulation signs after stopping external chest compression can be maintained for more than 20 min. The disputes on the concept of ROSC are related to the time span of ROSC prediction model research. When Gräsner et al. [14] published the research on the prediction model of the ROSC after cardiac arrest (RACA) score in 2011, the academic community had not reached a consensus on sustained ROSC. Until 2019, the Utstein Working Group no longer kept silent on this topic and said in the relevant statement that ROSC, as a core outcome element, was defined as the recovery of circulation without continuous chest external compression, that is, sufficient pulse/heart rhythm was recovered through palpation, auscultation, arterial blood pressure waveform, or systolic pressure greater than 50 mm·Hg, while sustained ROSC was considered as the ROSC duration greater than 20 min [24]. In view of the fact that the research on the ROSC prediction model is still under development and improvement and the concept of major outcome events has not yet reached an agreement, clinical doctors and nurses should pay attention to the application range of ROSC as the major outcome event when selecting the reference prediction model. Moreover, it is suggested that the definitions of ROSC and sustained ROSC should be consistent with the latest international consensus when constructing and developing the ROSC prediction model applicable to native CA patients.

### 4.3. Analysis of Model Predictors

Although the predictive factors of ROSC in OHCA patients vary in different models, there are still some commonalities. Among them, patient factors include age, gender, etiology, and initial heart rhythm, while external factors include EMS arrival time/BLS intervention time, location, bystander CPR, witnessed during sudden arrest, and ACLS duration/compression duration. Demographic characteristics based on age and gender are generally considered to be closely related to ROSC. The probability of cardiovascular disease and the risk of OHCA increase with age. The elderly tend to have a lower success rate of ROSC after resuscitation due to organic weakness and basic comorbidity. In particular, it is worth noting that age 75 may be an inflection point, with a linear decline in 30-day survival with up to age 75 and a more significant slope after age 75 [25]. Male is considered a risk factor in most models, which is mainly related to less estrogen in men. Although the mechanism of action is still unclear, estrogen does have a certain protective effect on the heart and nerves of CA patients, so women show a survival benefit in early ROSC and 1.26 times higher 1-year survival rate than men [26]. The ROSC rate of OHCA induced by different etiologies is also different, and the etiologies of OHCA are generally classified into 5H (hypoxemia, hypothermia/hyperthermia, hypokalemia/hyperkalemia, hypovolemia, and hypoglycemia/hyperglycemia) and 5T (tablets, tamponade, thrombosis, tension pneumothorax, and toxins); in contrast, cardiogenic OHCA can often be intervened by drugs, defibrillation, and interventional procedures in the prodromal, onset, and arrest stages, and ROSC is easier to achieve in the prime time [19]. The initial rhythm type of OHCA patients can be divided into defibrillable rhythm and nondefibrillable rhythm. For patients with defibrillable rhythm such as ventricular fibrillation or pulseless ventricular tachycardia, the first witness can obtain AED in public places to defibrillate them so as to increase the probability of successful resuscitation. On the contrary, when the initial rhythm of OHCA patients is nondefibrillable rhythm such as ventricular arrest, pseudoelectromechanical dissociation, and ventricular escape, the administration of electric shock will aggravate the myocardial injury [14]. External factors seem to be more important for OHCA patients than personal factors. Since OHCA needs CPR within 4 minutes, the location of the patient when CA occurs, whether it is witnessed or whether the bystander performs CPR, and the time of chest compressions are critical to whether the patient can be found and rescued at the first time. The arrival time of EMS and the duration of ACLS can help the patient enter the next link of the life chain as soon as possible and obtain continuous advanced life support, thereby improving the ROSC probability. In addition, the model results of Kim et al. [16] showed that partial pressure of blood oxygen (PO_2_) and base excess (BE) can also predict ROSC in OHCA patients, which has not been mentioned by other models. It is generally believed that the death of OHCA patients is closely related to hypoxic brain damage and hypoxemia, and ensuring PO_2_ of patients has a positive significance in improving the ROSC rate and neurological prognosis of OHCA patients. However, some studies have shown that there is no significant relationship between the survival rate of OHCA patients and PO_2_. Therefore, it is still controversial whether PO_2_ is related to the ROSC rate of OHCA patients [27]. In addition, base excess can reflect the degree of systemic tissue acidosis, the lower the value of base excess, the higher the risk of mortality and coagulation disorders of patients, and should be continuously monitored during resuscitation [28]. However, there is not enough evidence to show that base deficit can be used as a predictor of ROSC. Moreover, due to the limitations and deficiencies of this model in performance reporting and external verification, the predictive value of PO_2_ and BE still needs to be further verified. The model of Liu et al. [21] demonstrated that administration before admission is a positive predictor, which is consistent with the recommendations of AHA guidelines. According to AHA guidelines, the early task for OHCA patients is to achieve ROSC as soon as possible. Adrenaline, as the preferred rescue drug, can improve the success rate of ROSC by improving myocardial blood supply, cerebral perfusion, bronchiectasis, and other mechanisms [29].

As a special branch of OHCA, TOHCA is usually triggered due to hemorrhagic shock, hypoxia, tension pneumothorax, or pericardial tamponade after severe trauma. Therefore, its survival rate is significantly lower than that of cardiogenic OHCA. Emerging evidence has suggested that improving the survival rate of TOHCA contributes to the early ROSC rate [30, 31]. Among the included studies, only the study of Kuo et al. [20] used TOHCA patients as subjects to develop TOHCA scores for predicting ROSC failure. Obvious chest injury, body temperature below 33°C, and possible etiologies of OHCA are independent risk factors for ROSC failure after 45 minutes of CPR [20]. Obvious chest injury is often accompanied by tension pneumothorax and post-traumatic asphyxia, and its treatment requires a professional doctor to carry out reversible primary disease and surgical thoracotomy. Therefore, traditional chest compression and artificial respiration by ordinary first witnesses outside the hospital have little effect on TOHCA patients, even deteriorate the disease, and reduce the success rate of ROSC [32]. Although hypothermia therapy before ROSC has a protective effect on the neurological prognosis of OHCA patients, whether it is applicable to TOHCA patients with existing hypothermia is still controversial [33, 34]. When the core temperature is lower than 35°C, the body function will continue to decline, leading to respiratory failure, heart failure, and renal failure until CA attacks [34]. TOHCA patients with hypothermia are often accompanied by complications such as coagulation dysfunction and acidosis, which form the triad of traumatic lethality, further deteriorate the functions of various organs, and sharply increase the mortality rate [35]. In addition to trauma, the presence of other potential causes of OHCA, such as poisoning, sepsis, COVID-19 infection, allergy, drowning, chronic obstructive pulmonary disease (COPD), hyperkalemia, and hypokalemia, makes the ROSC rate of TOHCA patients more dismal [8, 36]. The TOHCA score can be employed as a reference tool to help clinical decision makers deal with the ethical conflicts caused by limited medical resources and ensure that medical resources can be invested as early as possible from patients who still end up with ROSC failure after 45 minutes of CPR to other patients with a higher probability of ROSC success. However, considering that giving up a rescue for TOHCA patients may cause medical staff to fall into a moral dilemma and medical disputes, it is suggested that the clinical application of this score should be cautious.

For the development of the IHCA prediction model, only the study of Harrison et al. [15] met the inclusion criteria. Like for OHCA patients, age, gender, and initial heart rhythm are also predictors of ROSC for IHCA patients. In addition, predictors of ROSC in IHCA patients also include the reason for the visit, length of hospital stay, and location of IHCA [15]. The reason for the patient's visit is closely related to the primary disease. Patients with coronary heart disease, myocardial infarction, and other cardiogenic diseases and/or respiratory diseases have a higher risk of IHCA, and they are more difficult to achieve sustained ROSC than other patients because of the organic and functional changes caused by the primary disease [37]. As indicated by Tran et al. [38] and Harrison et al. [39], with the prolongation of hospital stay, the frequency of IHCA is higher and the prognosis after resuscitation is worse. If the patients are accompanied by the deterioration of other diseases during their hospital stay, the probability of IHCA after resuscitation and the risk of ROSC failure will increase. The location of IHCA also affects the success rate of ROSC. The ROSC success rate of IHCA occurring in the emergency department, intensive care unit (ICU), and cardiology department is higher than that in other departments [40]. Different locations in the hospital also lead to different arrival times of the rapid response team (RRT), thus affecting ROSC [41].

### 4.4. Strength and Limitations

To our knowledge, this is the first study to comprehensively analyse and assess a predictive model for the return of spontaneous circulation in cardiac arrest patients. Prior to conducting our study, we conducted research plans and information registries, as well as normative studies and reports using the Cochrane Handbook and CHARMS.

Now also, we cannot rule out the possibility that our study has limitations. At the outset, the pooled AUC is based on the standard error, while some studies do not directly provide this indicator, and there is no other method to synthesize the AUC data from the indicators existing in the original study. Therefore, the pooled AUC can only be calculated by indirect inference of the standard error, which affects the accuracy of the results to a certain extent. In addition, not all studies reported the evaluation indicators such as sensitivity, specificity, PPV, and NPV of the prediction model, so we only performed a meta-analysis on the AUC, sensitivity, and specificity of the models with some included indicators and available indicators. Second, considering that the medical treatment of children, pregnant women, and other special groups is different from that of adults, this study only includes the ROSC prediction model whose research objects are 18 years or older but it is still important to develop the ROSC prediction model for special groups. Finally, we only tested prediction models for Chinese and English databases, so there may be other language prediction models that we missed.

## 5. Conclusion

This study includes eight prediction models for ROSC, including OHCA, TOHCA, and IHCA, all of which report good discriminative performance. Unfortunately, these models have a high risk of bias and a large difference in the overall performance. Thus, the external verification of multicenter is still needed before the practical application. Further studies aimed at calibrating and optimizing the current model based on the actual situation or constructing a more standardized ROSC prediction model in strict accordance with the PROBAST evaluation criteria so as to improve the accuracy and practicability of the model and support its clinical application after publication.

## Figures and Tables

**Figure 1:** PRISMA diagram.

**Figure 2:** Summary of predictors present in the included OHCA models.

**Figure 3:** Forest plot of the pooled AUC for the ROSC model in meta-analysis.

**Figure 4:** Forest plot of the pooled sensitivity for the ROSC model in meta-analysis.

**Figure 5:** Forest plot of the pooled specificity for the ROSC model in meta-analysis.

**Table 1:** Basic characteristics of the ROSC prediction model included.

Authors and years	Country	Object	Sample (missing data)	Data sources	ROSC rate (%)	Candidate variables' number	Variable selection	Method	Validation	Model performance		Predictors in the final model
										AUC/C-index	Calibration	
Gräsner et al. [14] 2011	Germany	OHCA	7689 (1112)	GRR	43.8	9	Multivariate analysis was performed after univariate analysis	LR	Internal	0.710^1^	None	Sex, age, etiology, first witness identity, location, initial heart rhythm, bystander CPR, EMS arrival time
										0.731^2^		

Harrison et al. [15] 2014	UK	IHCA	24136 (<0.3%)	NCAA	45.0	7	Backward stepwise selection method	LR	Internal, external	0.733^*∗*^^1^	HL test, calibration plot, Cox calibrated regression, Brier scores	Age, sex, length of hospital stay, medical reasons, location, initial heart rhythm
										0.720^*∗*^^2^		
										0.725^*∗*^^3^		

Kim et al. [16] 2017	Korea	OHCA	727 (97)	ED	55.7	11	Multivariate analysis was performed after univariate analysis	Cox	Internal	None	Grønnesby and Borgan goodness of fit tests	Age, location, etiology, initial heart rhythm, time of BLS, prehospital low blood-flow time, PO_2_, ACLS duration, BE

Amnuaypattanapon et al. [17] 2020	Thailand	OHCA	347 (37)	ED	36.3	14	Backward stepwise selection method	LR	Internal	0.775^1^	None	Witnessed at arrest, time of BLS, CPR duration

Baldi et al. [18] 2020	Italy and Switzerland	OHCA	2709 (1224)	Pavia CARE and TiReCa	P: 16.9 T: 33.5	7	Multivariate analysis was performed after univariate analysis	LR	Internal, external	0.83^1^	None	Age, location, witnessed at arrest, bystander CPR, EMS arrival time, initial heart rhythm
										0.82^2^		
										0.77^3^		

Ji et al. [19] 2021	UK	OHCA	32789 (1817)	NHS	25.0	8	Multivariate analysis was performed after univariate analysis	MEM	Internal	0.70^1^	HL test, Cox calibration, Brier scores	Sex, bystander CPR, etiology, initial heart rhythm
										0.67^2^		

Kuo et al. [20] 2022	China	TOHCA	580 (10)	A trauma center in Taiwan	21.4	13	Multivariate analysis was performed after univariate analysis	LR	Internal, external	0.662^1^	None	Obvious chest injury, body temperature below 33°C, and possible etiology of OHCA

Liu et al. [21] 2022	Singapore	OHCA	170678 (9146)	PAROS	8.26	13	The importance of the candidate predictors was ranked and the top five variables were included	RF	Internal	0.715^1^	None	Age, witnessed at arrest, EMS arrival time, initial heart rhythm, prehospital administration
										0.806^2^		

ROSC: recovery of spontaneous circulation; OHCA: out-of-hospital cardiac arrest; IHCA: hospital cardiac arrest; TOHCA: traumatic out-of-hospital cardiac arrest; ED: emergency department; GRR: German recovery registration system; NCAA: The UK's National Cardiac Arrest Audit; Pavia CARE: Pavia department cardiac arrest registration system; TiReCa: Ticino Regional Cardiac Arrest Registry; NHS: National Health Service; PAROS: the Pan-Asian recovery outcome registry. ^1^: development result, ^2^: internal validation result, ^3^: external validation result; AUC: area under the curve; C-index: concordance index; ^*∗*^: consistency index result; HL test: Hosmer–Lemeshow test; LR: logistic regression; Cox: Cox regression model; MEM: mixed-effect model; RFs: random forests; CPR: cardiopulmonary resuscitation; EMS: emergency medical services; BLS: basic life support; ACLS: advanced cardiac life support; PO_2_: partial pressure of blood oxygen; BE: base excess.

**Table 2:** Bias risk assessment results included in the mode (PROBAST evaluation results).

First authors	Risk of bias				Applicablity			Overall	
	Participants	Predicators	Outcome	Analysis	Participants	Predicators	Outcome	Risk of bias	Applicablity
Gräsner et al. [14]	Low	Low	Low	High	High	High	High	High	High
Harrison et al. [15]	Low	Low	Low	High	High	High	High	High	High
Kim et al. [16]	High	Low	Low	High	High	High	High	High	High
Amnuaypattanapon et al. [17]	Low	Low	Low	High	High	High	High	High	High
Baldi et al. [18]	Low	Low	Unclear	High	High	High	High	High	High
Ji et al. [19]	Low	Low	Unclear	High	High	High	High	High	High
Kuo et al. [20]	High	Low	Low	High	High	High	High	High	High
Liu et al. [21]	Low	Low	Unclear	High	High	High	High	High	High

## Data Availability

The models' data supporting this systematic review are from previously reported studies and datasets, which have been cited. These prior studies are cited at relevant places within the text as references [14–21]. The processed data are available within the article.
